The article "The Diagnostic Value of Serum GDF15 and hs-CTnT in Elderly Patients with Acute Myocardial Infarction" was retracted in 2023. Reasons: unreliable results or conclusions; concerns about the data; concerns about the peer review; concerns about the citations.

# The Diagnostic Value of Serum GDF15 and hs-CTnT in Elderly Patients with Acute Myocardial Infarction

**DOI:** 10.1155/2022/9281636

**Published:** 2022-05-20

**Authors:** Yejun He, Hui Wang, Zhihua Fang

**Affiliations:** ^1^Department of Special Examination, The First People's Hospital of Fuyang District, Hangzhou 311400, China; ^2^Department of Pathology, The First People's Hospital of Fuyang District, Hangzhou 311400, China; ^3^Department of Public Health, Dayuan Community Health Service Center, Fuyang District, Hangzhou 311400, China

## Abstract

**Objective:**

To analyze the diagnostic value of serum growth differentiation factor 15 (GDFl5) and high-sensitivity troponin T (hs-cTnT) in elderly acute myocardial infarction (AMI).

**Methods:**

A retrospective analysis of 165 patients with acute chest pain admitted to the Department of Cardiology in our hospital from January to December 2020, Among them, 76 AMI patients (AMI group), 89 non-AMI patients (non-AMI group), and 80 healthy people were selected as the control group during the same period. Compare the three groups of serum GDF15, hs-CTnT levels, and left ventricular ejection fraction (LVEF) parallel correlation analysis, and draw the receiver operating curve (ROC) of serum GDF15 and hs-CTnT levels to diagnose AMI.

**Results:**

The serum GDF15 and hs-CTnT levels of the AMI group were significantly higher than those of the non-AMI group and the control group, and the difference was statistically significant (*p* < 0.01). The LVEF was significantly lower than the non-AMI group and the control group, whose difference was statistically significant (*p* < 0.01). Among them, the indicators of the non-AMI group were both higher and lower than the control group, and the difference was statistically significant (*p* < 0.01). Serum GDF15 and hs-CTnT levels of AMI patients increased with the increase of NYHA grade, among which grade IV group was significantly higher than grade I∼II group and grade III group (*P* < 0.01), and grade III group was significantly higher than grade I∼II Group (*p* < 0.01). Pearson correlation analysis showed that GDF15 and hs-CTnT levels of AMI patients were significantly negatively correlated with LVEF (*r* = −0.584, −0.612, − < 0.01). The ROC curve showed that GDF15 had a high specificity (93.75%) and hs-CTnT has a high sensitivity (90.67%). The area under the curve for diagnosing AMI is > 0.7 (0.895, 0.948). The sensitivity of the combined detection and the specificity are higher than that of individual detection.

**Conclusion:**

Serum GDF15 and hs-CTnT are highly expressed in elderly patients with AMI. The combined detection of the two can improve the efficiency of AMI diagnosis. GDF15 can be used as a new biomarker for AMI diagnosis and disease monitoring.

The article "The Diagnostic Value of Serum GDF15 and hs-CTnT in Elderly Patients with Acute Myocardial Infarction" was retracted in 2023. Reasons: unreliable results or conclusions; concerns about the data; concerns about the peer review; concerns about the citations.

## 1. Introduction

Acute myocardial infarction (AMI) is the most serious fatal disease in the cardiovascular system of the elderly. It is caused by a variety of internal and external environmental factors such as previous diseases, lifestyle, mood, and weather changes and causes the blockage of the blood supply channel of the heart, resulting in the imbalance of coronary artery oxygen supply and demand, which lead to myocardial necrosis, heart failure, and even death [1]. The main symptoms of AMI are severe and persistent compressive pain in the anterior heart area or pain in the retrosternum, accompanied by feelings of suffocation or near death. Factors that induce thrombosis and coronary artery obstruction can cause disease [2]. Its morbidity and mortality are high, and timely treatment is the key to save the lives of patients. However, some patients have atypical symptoms and no strong sense of pain. Heart failure or shock symptoms occur immediately after onset, which is easy to be missed and misdiagnosed, increasing the risk of death [3]. Therefore, finding the key detection indicators of AMI has important guiding significance for the realization of early diagnosis [4].

It was found that serum high-sensitivity troponin T(hs-CTnt) is a key biomarker of myocardial injury and has a higher sensitivity than ordinary cardiac troponin. Although it is an indispensable means for the early diagnosis and elimination of AMI, single indicator detection still has the limitations of missed diagnosis and misdiagnosis [5]. Other studies have found that growth differentiation factor-15 (GDF-15) has been proved to be abnormally expressed in metabolic diseases, cardiovascular diseases (atherosclerosis, chronic heart failure, coronary heart disease, etc.), malignant tumors, and other diseases. As a member of the tumor necrosis factor-superfamily (TGF-*β*), it is the only hormone activated when the body is under acute or long-term stress and plays a biological function by regulating related pathways, so it can be attempted as a potential biomarker for the early diagnosis of AMI [6]. The combined diagnosis of hs-CTnt and GDF-15 in AMI has not been reported so far. To analyze the diagnostic value of GDFl5 and hs-cTnT in elderly AMI, in this study, real-time fluorescence quantification (RT-PCR) and enzyme-linked immunosorbent assay (ELISA) were used to detect the expression levels and diagnostic value of the two methods in AMI. Through our research, GDF15 can be widely used as a new biomarker for the diagnosis and monitoring of AMI.

## 2. Data and Methods

### 2.1. General Information

This study, approved by the Medical Ethics Committee of our hospital, retrospectively, analyzed 165 patients with acute chest pain as the main symptom admitted to the Department of Cardiology of our hospital from January to December 2020. There were 76 AMI patients (AMI group) and 89 non-AMI patients (non-AMI group). The disease types of non-AMI group were arrhythmia 20 cases, unstable angina 33 cases, pleurisy 12 cases, heart failure 18 cases, and pulmonary embolism 6 cases. In the AMI group, according to the New York Heart Association Cardiac Function Classification (NYHA classification) [7], there were 24 cases of grade I ∼ II, 21 cases of grade III, and 30 cases of grade IV. Inclusion criteria: (1) all patients met the diagnostic criteria of AMI in guidelines for diagnosis and treatment of acute myocardial infarction [8], and all patients met the diagnostic criteria of non-AMI group in the 9th edition of internal medicine [9] and were confirmed by coronary angiography, electrocardiogram, chest X-ray, cardiac ultrasound, etc.; (2) all patients had the first onset and normal coagulation function; (3) 60 to 79 years old.

The article "The Diagnostic Value of Serum GDF15 and hs-CTnT in Elderly Patients with Acute Myocardial Infarction" was retracted in 2023. Reasons: unreliable results or conclusions; concerns about the data; concerns about the peer review; concerns about the citations.

Exclusion criteria: (1) patients with other cardiovascular diseases (such as viral myocarditis, old myocardial infarction, and cardiogenic shock) and cerebrovascular diseases; (2) a history of surgical treatment or severe trauma within 3 months; (3) patients with diseases of endocrine, blood system, and immune system; (4) patients with dysfunction of other vital organs.

During the same period, 80 healthy subjects were selected as the control group, and there was no statistical difference in the general data of the three groups (*p* > 0.05), indicating comparability (Table 1). All subjects were aware of the study and signed informed consent.

### 2.2. Detection Methods and Instruments

After enrollment, 5 ml of fasting venous blood was taken from all subjects in the morning and placed in a centrifuge at a rate of 3000 r/min for 10 min after standing for 2 h. After separation, the serum was taken for immediate detection or frozen storage at −20°C for testing.

Serum GDF‐15 levels were determined by enzyme-linked immunosorbent assay (ELISA). The serum hS-CTnt level was detected by automatic electrochemiluminescence immunoassay analyzer (model: Roche Elecsys 2010). The instrument and kit were purchased from Roche Diagnostic Products (Shanghai) Co., LTD. Serum hs-CTnt was normal between 0 ng/L and 0.15 ng/L. Serum GDF‐15 < 1200 ng/L was normal, >1800 ng/L was significantly elevated, and between the two was slightly elevated.

The above experimental steps are strictly in accordance with the instrument and kit instructions, and the same indicator should be operated by the same person. The left ventricular ejection fraction (LVEF) of all subjects was measured by a color Doppler ultrasound instrument purchased from Philips, the Netherlands, and the body mass index (BMI) of all subjects was calculated.

The article "The Diagnostic Value of Serum GDF15 and hs-CTnT in Elderly Patients with Acute Myocardial Infarction" was retracted in 2023. Reasons: unreliable results or conclusions; concerns about the data; concerns about the peer review; concerns about the citations.

### 2.3. Observation Indicators

(1) Serum levels of GDF15, hs-CTnt, and LVEF were compared among the three groups. (2) The levels of serum GDF15 and hs-CTnt in patients with different NYHA grades in the AMI group were compared. (3) Pearson correlation analysis of GDF15, hs-CTnt levels, and cardiac function in AMI patients. (4) The sensitivity, specificity, and diagnostic coincidence rate of serum GDF15 and hs-CTnt alone and combined detection of AMI were calculated.

### 2.4. Statistical Processing

SPSS 21.0 software was used to process all data collected in this study, and all measurement data parameters were expressed in the form of mean ± standard deviation (*X* ± *S*). Comparison between groups was performed by one-way ANOVA combined with post-Bonferroni test, denoted by F. Counting data were expressed in the form of case/percentage. Chi-square test and Chi-square split test were used for comparison between groups, denoted by Z. Pearson correlation was used for correlation analysis, and the receiver operating curve (ROC) was drawn to test the diagnostic value of serum GDF15 and hs-CTnt in AMI. Area under the curve >0.70 was considered to be of diagnostic value, and *p* < 0.05 was considered to be statistically significant.

## 3. Results

### 3.1. Comparison of Serum GDF15 and hs-CTnt Levels

Serum levels of GDF15 and hs-CTnt in the AMI group were significantly higher than those in non-AMI group and control group (*p* < 0.01), and LVEF was significantly lower than those in non-AMI group (*p* < 0.01), as shown in Table 2.

### 3.2. Comparison of Serum GDF15 and hs-CTnt Levels in Patients with Different NYHA Grades

Serum GDF15 and hs-CTnt levels in AMI patients increased with the increase of NYHA grade. The level IV group was significantly higher than the level i ∼ ii and III groups (*p* < 0.01), and the level III group was significantly higher than the level i ∼ ii groups (*p* < 0.01), as shown in Table 3.

### 3.3. Pearson Correlation Analysis between GDF15, hs-CTnt Levels, and Cardiac Function in AMI Patients

Pearson correlation analysis showed that GDF15 and hs-CTnt levels were significantly negatively correlated with LVEF in patients with AMI (*r* = -0.584, -0.612, *p* < 0.01).

### 3.4. ROC Curve of Serum GDF15 and hs-CTnt for AMI Diagnosis

Sensitivity, specificity, and area under ROC curve were 84.21%, 93.75%, and 0.895(95%CI: 0.842–0.948, *p* < 0.01) for GDF15 and 90.67%, 89.87%, and 0.948 for hs-CTNT (95%CI: 0.916–0.979, *p* < 0.01) and GDF15+ hs-CTnt 95.64%, 92.97%, and 0.963 (95%CI: 0.939–0.988, *p* < 0.01). The sensitivity, specificity, and diagnostic coincidence rate of the combined test were higher than those of single test, as shown in Figure 1.

The article "The Diagnostic Value of Serum GDF15 and hs-CTnT in Elderly Patients with Acute Myocardial Infarction" was retracted in 2023. Reasons: unreliable results or conclusions; concerns about the data; concerns about the peer review; concerns about the citations.

## 4. Discussion

Epidemiological data show that there are at least 500,000 new AMI patients in China every year, and the number of AMI deaths worldwide is more than 8.5 million, which is more than 50% of the total death rate of cardiovascular diseases [10]. Patients with AMI usually present with acute and persistent severe chest pain, which is confirmed by electrocardiogram and serological examination. 3∼6 h after chest pain is the best time for reperfusion therapy to control AMI mortality. Early diagnosis and early treatment are very important. The selection of serological indicators is directly related to the diagnostic efficiency of AMI [11]. In this study, serum GDF15 and hs-CTnt were selected to demonstrate their expression and diagnostic value in AMI.

The results of this study showed that the levels of SERUM GDF15 and hs-CTnt in the AMI group were significantly higher than those in the non-AMI group and the control group, and LVEF was significantly lower than those in the non-AMI group and the control group. The levels of serum GDF15 and hs-CTnt in patients with AMI increased with the increase of the NYHA grade. Pearson correlation analysis showed that GDF15 and hs-CTnt levels were significantly negatively correlated with LVEF, which proved that serum GDF15 and hs-CTnt levels were highly expressed in AMI patients. The higher the cardiac function grade is, the more serious the degree of myocardial injury is, and the higher the expression of both levels is. Therefore, the determination of GDF‐15 and hs-CTnt in patients with AMI is helpful for early diagnosis and evaluation of disease development. Because (1) GDF-15 affects the expression of a variety of signaling pathways, only a small amount of it exists in placental tissue under normal physiological state, and low expression is observed in kidney and pancreas tissues, while high expression is observed in the disease state [12]. GDF-15 protein is involved in the evolution of cardiovascular diseases, and its expression is elevated in the pathological process of such diseases. GDF-15 protein regulates myocardial injury by binding to TGF-*β* receptors on the surface of cardiomyocytes and then activates SMAD and other pathways. Cardiomyocytes of patients in the AMI state are continuously damaged, and GDF-15 is induced to present an elevated state [13]. On the contrary, the higher cardiac function grading is, the more likely it is to damage cardiac hemodynamic force and myocardial cell membrane, while increasing cardiac load, elongating myocardial fibers, and stimulating excessive release of myocardial injury markers. Therefore, the higher the NYHA grade, the more severe myocardial injury and the more obvious the serum GDF‐15 level expression; therefore, it can be used as a new biomarker for AMI diagnosis and disease monitoring [14]. (2) hs-CTnt expression can be abnormally high within about 3 h after the onset of AMI and can maintain an upward trend for more than 10d after myocardial necrosis. Therefore, the hs-CTnt value can increase according to the function classification, and dynamic monitoring can reflect the severity of AMI patients [15]. At the same time, hs-CTNI is an ideal marker of myocardial defect, which is abundant in myocardial tissue and has a long detection window. It plays an important role in evaluating the area of myocardial infarction, the effect of thrombolytic therapy, and the differential diagnosis of cardiological diseases with chest pain as the main symptom and has always been the “gold standard” in the diagnosis of myocardial injury [16].

The article "The Diagnostic Value of Serum GDF15 and hs-CTnT in Elderly Patients with Acute Myocardial Infarction" was retracted in 2023. Reasons: unreliable results or conclusions; concerns about the data; concerns about the peer review; concerns about the citations.

We further drew ROC curves and found that GDF15 had a higher specificity than hs-CTnt (93.75% vs. 89.87%), and the sensitivity of hs-CTnt was higher than GDF15 (90.67% vs. 84.21%), and the area under curve for the diagnosis of AMI was greater than 0.7 (0.895, 0.948). The sensitivity and specificity of combined detection were higher than those of single detection, confirming the clinical application value of the two methods in the diagnosis of AMI. At the clinical stage, it has been confirmed that hs-CTNT has better detection accuracy than other biomarkers, and it can reflect the minor damage of myocardial tissue and is the primary diagnostic marker of AMI [17]. At present, there are not many clinical reports on the detection of hs-CTnt combined with other markers of myocardial injury, and the results of combined detection can obtain high sensitivity and low specificity. This may be related to other factors such as susceptibility of other markers of myocardial injury to other diseases and inconsistent detection time window. Therefore, GDF15 with high specificity was selected in this study to obtain ideal sensitivity and specificity values (95.64% and 92.97%). Wu and Guo [18] showed that GDF-15 may be involved in ventricular remodeling in patients with AMI-induced heart failure and is related to the severity of heart failure. Zhang et al. [19], 20 pointed out that GDF-15 was significantly correlated with the size of myocardial infarction in patients with AMI and could be used as a marker of myocardial infarction. The results of this study confirmed that GDF-15 can be used for the early diagnosis of AMI in clinical practice, and its limitations of strong specificity and low sensitivity can be consolidated and improved by combining hs-CTnt diagnosis. However, the clinical understanding of GDF-15 is only at the initial stage, and the specific pathogenic mechanism of GDF-15 in AMI still needs to be further clarified, and a large number of in-depth studies are needed in the later stage. It is noteworthy that hs-CTnt has a high diagnostic sensitivity for AMI. However, due to the imbalance between supply and demand of blood in the body, the hs-CTnt index in some patients with non-AMI diseases, such as chronic heart failure and diabetes, is still higher than the upper limit of the normal range, so as to increase the false positive rate of such non-AMI patients. Therefore, the specificity should be combined with the comprehensive situation of patients in clinical practice.

The article "The Diagnostic Value of Serum GDF15 and hs-CTnT in Elderly Patients with Acute Myocardial Infarction" was retracted in 2023. Reasons: unreliable results or conclusions; concerns about the data; concerns about the peer review; concerns about the citations.

## 5. Conclusion

In conclusion, serum GDF15 and hs-CTnt are highly expressed in elderly patients with AMI, and their combined detection can improve the diagnostic efficiency of AMI. GDF15 can be widely used as a new biomarker for the diagnosis and monitoring of AMI in clinical practice.

## Figures and Tables

**Figure 1:** ROC curve of serum GDF15 and hs-CTnt for AMI diagnosis.

**Table 1:** Comparison of general data of the three groups of subjects.

Group		Gender (male/female, example)	Average age (years)	Average BMI (kg/m^2^)

Group AMI	Cardiac function grade i ∼ ii (*n* = 24)	16/8	71.17 ± 9.93	23.56 ± 2.77
	Cardiac function grade iii (*n* = 22)	14/8	72.62 ± 10.35	23.19 ± 2.42
	Cardiac function grade iv (*n* = 30)	20/10	72.94 ± 8.80	24.07 ± 2.84
Non-AMI group (*n* = 89)		54/35	71.33 ± 10.19	23.62 ± 2.72
Control group (*n* = 80)		50/30	70.48 ± 8.93	23.18 ± 2.63
F value		0.731	0.117	0.097
*p* values		0.948	0.907	0.886

**Table 2:** Comparison of serum GDF15 and hs-CTnt levels ($\bar{x}$ ±*s*).

Group	GDF15 (ng/L)	hs-cTnT (ng/L)	LVEF (%)
Control group (*n* = 80)	573.39 ± 67.42	0.014 ± 0.003	64.77 ± 5.48
Non-AMI group (*n* = 89)	1913.73 ± 101.55	0.217 ± 0.018	50.13 ± 4.62
AMI group (*n* = 76)	3328.46 ± 168.45	0.753 ± 0.037	44.72 ± 5.31
*F*	105.444	208.079	31.742
*p*	0.000	0.000	0.000

**Table 3:** Comparison of serum GDF15 and hs-CTnt levels in patients with different NYHA grades ($\bar{x}$ ±*s*).

NYHA classification	GDF15 (ng/L)	hs-cTnT (ng/L)
I∼II(*n* = 24)	2643.62 ± 135.88	0.458 ± 0.028
III (*n* = 22)	3253.79 ± 156.34	0.677 ± 0.035
IV (*n* = 30)	3574.82 ± 178.95	0.815 ± 0.057
*F*	142.788	41.463
*p*	0.000	0.000

## Data Availability

The data used to support the findings of this study are available from the corresponding author upon request.
